# Effect of Warming Yang, Tonifying Kidney, and Removing Arthralgia Therapy on Cold-Dampness Arthralgia Type Ankylosing Spondylitis and Its Influence on the Levels of Humoral Factor in Human Serum

**DOI:** 10.1155/2022/8348272

**Published:** 2022-05-09

**Authors:** Jing Li

**Affiliations:** Affiliated Hospital of Hubei University of Traditional Chinese Medicine, Hubei Hospital of Traditional Chinese Medicine, Wuhan, Hubei 430060, China

## Abstract

**Objective:**

This study is aimed at exploring the effect of warming Yang, tonifying kidney, and removing arthralgia therapy in the treatment of cold-dampness arthralgia type ankylosing spondylitis (AS) and the effects on the levels of humoral factor in human serum*. Method.* A total of 72 patients with cold-dampness arthralgia type AS treated in our hospital from May 2020 to June 2021 were selected and divided into the observation group (*n* = 36) and control group (*n* = 36) according to the random number table method. The clinical efficacy of the two groups was observed. The traditional Chinese medicine (TCM) syndrome scores and clinical signs of the two groups were compared, and the pain situation of the two groups was evaluated by visual analog scale (VAS). Bath Ankylosing Spondylitis Disease Activity Index (BASDAI) and Bath Ankylosing Spondylitis Functional Index (BASFI) were used to evaluate the spinal function and activity of the two groups, and the levels of CXC-type chemokine ligand 16 (CXCL16), Dickkopf-1(DKK-1), interleukin-17 (IL-17), tumor necrosis factor-*α* (TNF-*α*), sclerostin (SOST) ,and bone morphogenetic protein 2(BMP-2) in serum of the two groups were measured.

**Results:**

The total effective rate of the observation group (91.67%) was significantly higher than that of the control group (66.67%) (*P* < 0.05). After treatment, the degree of improvement in TCM syndrome score, clinical signs, VAS score, BASDAI, BASFI, and the levels of CXCL16, TNF-*α*, IL-17, DKK-1, SOST, and BMP-2 in the observation group were significantly higher than that in the control group (all *P* < 0.05)*. Conclusion.* Warming Yang, tonifying kidney, and removing arthralgia therapy had a good effect on the treatment of cold-dampness arthralgia type AS, and it could effectively improve the clinical symptoms and signs, relieve pain, improve spinal motion, and relieve inflammation of patients.

## 1. Introduction

Ankylosing spondylitis (AS) is a chronic joint disease. The progression of this disease is relatively insidious, and the continuous development may lead to pain and limited movement in waist and back, which may affect the large joints of patients' limbs and seriously affect their daily life [1, 2]. The treatment of this disease needs active and effective methods. Nonsteroidal anti-inflammatory drugs are often used to treat the disease. This method can improve the pain symptoms of patients to a certain extent but cannot delay the development of the disease. In addition, long-term use of this type of drugs can cause adverse reactions in patients, and recurrence is prone to occur after drug withdrawal. Traditional Chinese medicine (TCM) has rich experience in the treatment of osteoarthritis and can effectively relieve the clinical symptoms and pain of patients. AS belongs to the category of “heumatism” in TCM and is an intermingled asthenia and sthenia syndrome. The main pathogenesis of cold-dampness arthralgia type AS is insufficiency of kidney essence and deficiency of Yang qi. The evil gas of cold dampness invades the joints, ultimately leading to the pain in back and loin. Cold-dampness arthralgia type is a common syndrome type in AS, and the treatment method of warming Yang to nourish kidney and dissipating cold to dehumidify should be adopted. Human CXC-type chemokine ligand 16 (CXCL16) is a chemokine produced by defensive immune cells at the invaded site, and it can promote the migration and infiltration of leukocytes; it is expressed in a variety of inflammatory diseases and can be involved in the occurrence and development of inflammatory diseases [3]. Dickkopf-1 protein (DKK-1) not only exists in the flat bone but also is expressed in tubular bone cells, and its level is negatively correlated with bone mineral density [4]. Interleukin-17 (IL-17) is the main factor secreted by Th17 cells [5]. TNF-*α* is a common inflammatory factor, directly involved in the occurrence and development of AS. Both OST and BMP-2 are ossification regulators and can be used to evaluate spinal joint damage. SOST inhibits osteoblastogenesis. BMP-2 induces the expression of bone proteins. According to relevant studies, the level of Th17 cells in peripheral blood of patients with AS is increased significantly. The purpose of this study was to explore the effect of warming Yang, tonifying kidney, and removing arthralgia therapy in the treatment of cold-dampness arthralgia type AS and its effects on humoral factor levels, which are reported as follows.

## 2. Materials and Methods

### 2.1. General Data

A total of 72 patients with AS cold-dampness arthralgia syndrome treated in our hospital from May 2020 to June 2021 were selected and divided into the observation group and control group according to the random number table method, with 36 cases in each group. In the observation group, there were 10 males and 26 females. The average age was 50.25 ± 6.15 years, with a range of 40-58 years. The course of disease ranged from 1 to 9 years, with an average of 4.52 ± 1.28 years. In the control group, there were 13 males and 23 females. The average age was 51.13 ± 5.86 years, with a range of 42-57 years. The course of disease ranged from 8 months to 10 years, with an average of 4.16 ± 1.98 years. The general data of the two groups were comparable (*P* > 0.05). All patients enrolled in this study signed informed consent. This study was approved by the Hospital Ethics Committee.

### 2.2. Western Medicine Diagnostic Criteria

Referring to the AS standard revised by the American Rheumatology Association in 1984 [6], patients who meet any one of articles (4) and (1)–(3) are diagnosed as AS with cold-dampness obstruction syndrome: (1) low back pain, morning stiffness > 3 months, and the activity is improved while the rest does not improve; (2) lumbar sagittal and frontal plane movement is limited; (3) compared with normal subjects of the same age and gender, thoracic motion is lower; and (4) unilateral sacroiliac arthritis grades III ~ IV or bilateral sacroiliac arthritis grades II ~ IV.

### 2.3. Standard of TCM Syndrome Differentiation

According to the standards in Guidelines for Clinical Research of New Chinese Medicines [7], cold-dampness arthralgia type AS refers to the symptoms of stiffness and pain of waist and spine, which can be aggravated in case of cold and decreased in case of heat, light tongue, white fur, and stringy pulse.

### 2.4. Inclusion Criteria

The inclusion criteria were as follows: patients who (1) met both the diagnostic standards of western medicine and TCM syndrome differentiation standards, (2) with grade III ~ IV sacroiliac arthritis; (3) with age ≥ 18 years, (4) with no use of nonsteroidal anti-inflammatory drugs or drugs with the same efficacy as those used in this study within one week before enrollment, and (5) were volunteered to participate in this study.

### 2.5. Exclusion Criteria

The exclusion criteria were as follows: (1) patients with grade IV sacroiliac arthritis; (2) patients with serious complications; (3) patients with diseases such as metabolic bone disease, psoriasis, and acute trauma; (4) patients with serious organ dysfunction such as heart, liver, and kidney dysfunction; and (5) patients with severe endocrine diseases

### 2.6. Methods

The control group was treated with sulfasalazine enteric-coated tablets (Shanghai Xinyi Tianping Pharmaceutical Co., Ltd., SFDA approval number: H31020557,CHN), and the observation group was treated with warming Yang, tonifying kidney, and removing arthralgia therapy on the basis of the control group. The TCMs of 30 g of aconite, 20 g of cooked Rehmannia glutinosa and cassia twig, 15 g of notopterygium root, 15 g of Radix Paeoniae Alba, 15 g of Herba Epimedii, 15 g of Radix angelicae pubescentis, 15 g of Achyranthes root, 15 g of Coix seed, 10 g of parsnip, 10 g of Eucommia ulmoides, 10 g of antler gum, 6 g of licorice, 6 g of Ephedra, and 6 g of white mustard seed were selected. All the abovementioned drugs were decocted in water, 1 dose/d, and were taken in the morning and evening. Both groups were treated continuously for 3 months.

### 2.7. Observation Indices

(1) Clinical efficacy was as follows. (2) TCM syndrome score was as follows: TCM syndrome scoring was conducted according to Guidelines for Clinical Research of New Chinese Medicines [7] and *Traditional Chinese Medicine Diagnostics* [8]. Lumbosacral pain, morning stiffness, lumbosacral back pain, and lumbar spine activity limitation were scored. Asymptomatic score was 0; if the symptoms did not affect patients' life and patients have fewer activity restrictions, the score was 1; if the symptoms mildly affect patients' life and patients have activity restrictions, the score was 2; if the patients' condition worsens and life is seriously affected, the score was 3. The higher the score is, the more serious the symptoms. (3) Physical indicators were as follows: the physical indicators of the distance between the occipital and the wall, the distance between the finger and the ground, the interarch distance, the range of motion of the thoracic cavity, the range of motion of the spine, and Schober's test indexes before and after treatment were compared. (4) Pain and functional scores were as follows: visual analog scale (VAS) [9] was used to evaluate the pain degree of the two groups. The total score was 0-10, including mild pain (1-3 points), moderate pain (4-6 points), and severe pain (7-10 points). The higher the score, the more severe the pain symptoms were. Bath Ankylosing Spondylitis Disease Activity Index (BASDAI) [10] and Bath Ankylosing Spondylitis Functional Index (BASFI) [11] were used to evaluate the spinal function and activity of the two groups. BASDAI consisted of 6 questions, and self-assessment was carried out according to the 10 cm visual analogy scoring method. 0 points indicated no impact, while 10 points indicated extreme severity. The total score was 0-60 points. BASFI consisted of 10 items, which were self-rated by 10 cm visual analogy scoring. The two ends of the horizontal line were “easy” and “impossible,” respectively. The higher the score was, the more serious the situation was. The total score was 0-100 points. (5) Levels of serum CXCL16, tumor necrosis factor-*α* (TNF-*α*), and interleukin-17 (IL-17) were as follows: the fasting venous blood of 3-5 ml was taken from patients in a sterile environment and centrifuged at 3000 r/min at room temperature for 10 min, and the levels of CXCL16, TNF-*α*, and IL-17 in serum were determined by enzyme-linked immunosorbent assay. (6) Levels of serum DKK-1, sclerostin (SOST), and bone morphogenetic protein-2 (BMP-2) were as follows: serum DKK-1, SOST, and BMP-2 were determined by ELISA. (7) Safety was as follows.

### 2.8. Efficacy Evaluation Criteria

The curative effect was evaluated according to Guidelines for Clinical Research of New Chinese Medicines [7]. Clinical recovery was as follows: lumbosacral pain and morning stiffness disappeared, spinal activity was not restricted, erythrocyte sedimentation rate returned to normal, and X-ray examination showed significant improvement of bone disease; remarkably effective was as follows: the patient's lumbosacral pain was significantly relieved, morning stiffness disappeared, range of spinal motion increased, erythrocyte sedimentation rate was close to the normal level, and X-ray examination showed that the bone lesions were relieved; effective was as follows: the patient had relief of lumbosacral pain, mild morning stiffness, improved range of motion of the spine, decreased erythrocyte sedimentation rate, and X-ray indicated relief of bone disease; ineffective was as follows: patients with lumbosacral pain, morning stiffness symptoms and other signs, and related indicators did not improve and even aggravated. Here is the following formula: total effective rate = clinical recovery + remarkably effective + effective.

### 2.9. Statistical Analysis

SPSS 20.0 statistical software was used to analyze and process the data. Measurement data were expressed as ^−^*x* ± *s*, independent sample *t*-test was performed for intergroup comparison, and paired *t*-test was used for intragroup comparison before and after treatment. The counting data were expressed as frequency or constituent ratio, and *χ*^2^ test or Fisher exact probability method was used to compare the disordered classified data. *P* < 0.05 indicated that the difference was statistically significant.

## 3. Results

### 3.1. Comparison of Clinical Efficacy between the Two Groups

The total effective rate was 91.67% in the observation group and 66.67% in the control group, and the difference between the two groups was statistically significant (*P* < 0.05, Table 1).

### 3.2. Comparison of TCM Syndrome Score between the Two Groups

Before treatment, there were no significant differences in the scores of morning stiffness, lumbosacral pain, back pain, and lumbar spine activity limitation between the two groups (all *P* > 0.05). After treatment, the scores of morning stiffness, lumbosacral pain, back pain, and lumbar spine activity limitation decreased in both groups, and the scores in the observation group were significantly lower than those in the control group (all *P* < 0.05, Table 2).

### 3.3. Comparison of Physical Signs between the Two Groups

Before treatment, there were no significant differences in occipital wall distance, maxillary stalk distance, finger ground distance, thoracic motion range, lumbar motion range, and spinal motion range between the two groups (all *P* > 0.05). After treatment, the occipital wall distance, maxillary stalk distance, and finger ground distance were decreased in both groups, and the thoracic motion, lumbar motion, and spinal motion range were increased. The improvement degree of each index in the observation group was significantly greater than that in the control group (*P* < 0.05, Table 3).

### 3.4. Comparison of Pain and Function Scores between the Two Groups

Before treatment, there were no significant differences in VAS, BASDAI, and BASFI scores between the two groups (*P* > 0.05). After treatment, VAS, BASDAI, and BASFI scores were decreased in both groups, and the scores in the observation group were significantly lower than those of the control group (all *P* < 0.05, Table 4).

### 3.5. Comparison of CXCL16, TNF-*α*, and IL-17 Levels between the Two Groups

Before treatment, there were no significant differences in the levels of CXCL16, TNF-ɑ, and IL-17 between the two groups (all *P* > 0.05). After treatment, the levels of CXCL16, TNF-*α*, and IL-17 in both groups were decreased, and the levels in the observation group were significantly lower than those in the control group (all *P* < 0.05, Table 5).

### 3.6. Comparison of Serum DKK-1, SOST, and BMP-2 Levels between the Two Groups

Before treatment, there were no significant differences in the levels of DKK-1, SOST, and BMP-2 between the two groups (all *P* > 0.05). After treatment, the levels of DKK-1 and BMP-2 in both groups decreased, while the levels of SOST increased. The improvement degree of each index in the observation group was greater than that in the control group, with statistical significance (*P* < 0.05, Table 6).

### 3.7. Comparison of Drug Safety between the Two Groups

There were no statistical significances in adverse reactions between the two groups (all *P* > 0.05, Table 7).

## 4. Discussion

Ankylosing spondylitis (AS) belongs to the category of “heumatism” in TCM. The pathogenesis of this disease is Yang qi deficiency and cold evil invasion. Cold dampness invasion of joints will lead to pain in the back and loin. According to the TCM theory, the kidney is the origin of the congenital essence, in charge of the bone and marrow. The back is Yang, which belongs to the kidney. It is dominated by the governor meridian and manages the circulation of Yang qi. The main pathogenesis of AS patients is congenital loss of support or insufficient endowment. Patients can show governor meridian cold and kidney deficiency. External pathogens invade the body, and the accumulation of pathogens can transform into cold, which is hidden in the back vein, leading to qi stagnation, blood stasis, and adverse activity of tendons and bones. Moreover, due to deficiency of kidney essence and deficiency of Yang qi in patients, the water and liquid metabolism in the body become imbalance. Then, blood stasis and phlegm turbidity are produced in the body, lead to blockage of the meridians, flow in the spine joints, and eventually cause AS. The external manifestation of AS is blood stasis and phlegm turbidity. The external reason is the invasion of external pathogens, and the internal reason is kidney deficiency and governor meridian cold. Therefore, the clinical treatment of this disease should be based on warming Yang and tonifying kidney, and then the treatment method of removing arthralgia and activating meridians is adopted to regulate the qi in the body. In this study, the method of warming Yang, tonifying kidney, and removing arthralgia used cooked Rehmannia glutinosa, antler gum, and aconite as the sovereign drugs, which has the effects of tonifying kidney, nourishing essence, reviving Yang and relieving adverse effects, dispelling cold, and relieving pain. Radix Paeoniae Alba, cassia twig, Herba Epimedii, and Achyranthes root were used as the ministerial drugs. Cassia twig has the effect of warming Yang and eliminating arthralgia; Radix Paeoniae Alba can soften the liver, relieve pain, nourish blood, and retaining Yin; Herba Epimedii can warm Yang; Achyranthes root has the function of tonifying liver and kidney and strengthening muscles and bones. The adjuvant drugs were notopterygium root, Radix angelicae pubescentis, Eucommia ulmoides, parsnip, Coix seed, and Ephedra. Notopterygium root can relieve rheumatic pains and dehumidify and dredge joints; Radix angelicae pubescentis can dispel rheumatism, removing arthralgia and relieving pain; A and B used together have the effect of dispelling rheumatism, dispersing cold and relieving pain. Coix seed can eliminate rheumatism and strengthen the spleen; Eucommia ulmoides can reinforce the liver and kidney; parsnip can dispel rheumatism and retaining moisture; white mustard seed can dredge collaterals and benefit qi; Ephedra has the function of warming and dispersing cold; licorice can mediate all the drugs. All drugs used together have the effects of dispelling rheumatism, dispersing cold and relieving pain. Modern pharmacological studies show that aconitines in aconite can effectively inhibit inflammation and relieve body pain, and aconite polysaccharide can enhance body immunity [12]; cooked Rehmannia polysaccharide can enhance immunity of the human body [13]; total glucosides of Radix Paeoniae Alba have analgesic and antispasmodic effects and can effectively inhibit inflammation [14]; cinnamaldehyde in cassia twig has analgesic and sedative effects [15]; epimedium can promote the proliferation and viability of osteoblasts [16]; decoction of notopterygium root and Radix angelicae pubescentis has anti-inflammatory and analgesic effects [17]; Eucommia ulmoides can promote the proliferation of osteoblasts [18].

In the present study, the control group was given conventional treatment, and the observation group was treated with the method of warming Yang, tonifying kidney, and removing arthralgia. The total effective rate of the observation group was 91.67%, higher than that of the control group (66.67%). After treatment, the improvement degree of TCM syndrome score, clinical signs, VAS, BASDAI, and BASFI scores in the observation group were superior to those in the control group, indicating that warming Yang, tonifying kidney, and removing arthralgia therapy can effectively improve the clinical symptoms and signs of AS patients, as well as their pain and spinal function. This may be related to the effects of aconite, Radix Paeoniae Alba, cassia twig, Herba Epimedii, prepared Rehmannia root, notopterygium root, and Radix angelicae pubescentis on inhibiting inflammation, enhancing immunity, and relieving pain. Previous studies have applied TCM in the treatment of AS cold-dampness obstruction, and the therapeutic effect is good [19]. The results of our study are consistent with that.

Human CXC-type chemokine ligand 16 (CXCL16) is a chemokine produced by defensive immune cells at the invaded site. It can promote the migration and infiltration of white blood cells, be expressed in a variety of inflammatory diseases, and participate in the occurrence and development of inflammatory diseases. Some studies believe that CXCL16 is involved in the pathogenesis of AS [20]. As a common inflammatory factor, TNF-*α* is directly involved in the occurrence and development of AS and closely related to the disease activity of AS [21]. Il-17 is a Th17 cell-secreted major factor newly discovered clinically in recent years. It is an early initiator of inflammatory response and can stimulate inflammatory response by promoting the release of inflammatory factors. After binding with receptors, IL-17 can act on the MAP kinase pathway to aggravate inflammatory response [22]. DKK-1 is a secreted glycoprotein, which can block Wnt signal transduction and inhibit cell proliferation and bone formation after binding with corresponding receptors. Its level is negatively correlated with bone mineral density and is highly expressed in the serum of AS patients [23]. Both SOST and BMP-2 are ossification regulators, which can be used to evaluate spinal joint damage. SOST inhibits osteoblast formation, while BMP-2 induces the expression of bone protein and promotes the formation of new bone. Under normal conditions, the two are in balance and antagonize each other, but if the balance is broken, the progression of AS can be accelerated [24, 25]. In the present study, the levels of CXCL16, TNF-*α*, IL-17, DKK-1, SOST, and BMP-2 after treatment in the observation group were improved more than those in the control group. These results indicated that the warming Yang, tonifying kidney, and removing arthralgia therapy could improve the inflammatory response and ossification factor more effectively in the treatment of AS. This may be related to the inhibitory effect of various TCMs in the warming Yang, tonifying kidney, and removing arthralgia therapy on the inflammatory response of the body, but the specific mechanism needs to be further explored. The comparison of drug safety between the two groups showed that there was no significant difference in the incidence of adverse reactions between the two groups, indicating that the warming Yang, tonifying kidney, and removing arthralgia therapy were safe in the treatment of AS, without aggravating the adverse reactions of patients while adding drugs.

In conclusion, the application of warming Yang, tonifying kidney, and removing arthralgia therapy in the cold-dampness arthralgia type AS could effectively improve the clinical symptoms and signs of patients, relieve their pain, improve their spinal mobility, relieve inflammatory response, and regulate the level of ossification factor, with good therapeutic effect. This therapy can be further applied in clinical practice.

## Figures and Tables

**Table 1:** Comparison of clinical efficacy between the two groups (cases (%)).

Group	Clinical recovery	Remarkably effective	Effective	Ineffective	Total effective rate
Observation group (*n* = 36)	13 (36.11)	16 (44.44)	4 (11.11)	3 (8.33)	33 (91.67)
Control group (*n* = 36)	6 (16.67)	10 (27.78)	8 (22.22)	12 (33.33)	24 (66.67)
*χ* ^2^					6.821
*P*					0.009

**Table 2:** Comparison of TCM syndrome score between the two groups (^−^*x* ± *s*, points).

Group	Morning stiffness score		Lumbosacral pain score		Low back pain score		Lumbar spinal mobility limitation score	
	Before treatment	After treatment	Before treatment	After treatment	Before treatment	After treatment	Before treatment	After treatment
Observation group (*n* = 36)	2.70 ± 0.51	1.38 ± 0.34^a^	2.69 ± 0.47	1.31 ± 0.79^a^	2.17 ± 0.51	0.81 ± 0.13^a^	2.08 ± 0.44	0.69 ± 0.67^a^
Control group (*n* = 36)	2.86 ± 0.35	1.81 ± 0.40^a^	2.67 ± 0.48	1.67 ± 0.48^a^	2.11 ± 0.32	1.06 ± 0.41^a^	2.06 ± 0.47	1.00 ± 0.41^a^
*t*	1.968	3.639	0.249	2.354	0.557	2.614	0.258	2.332
*P*	0.053	0.001	0.804	0.021	0.580	0.011	0.797	0.023

Note: compared with before treatment, ^a^*P* < 0.05.

**Table 3:** Comparison of physical signs between the two groups (^−^*x* ± *s*).

Group	Occipital wall distance (cm)		Maxillary stalk distance (cm)		Finger ground distance (cm)		Thoracic motion range (cm)		Lumbar motion range (cm)		Spinal motion range (°)	
	Before treatment	After treatment	Before treatment	After treatment	Before treatment	After treatment	Before treatment	After treatment	Before treatment	After treatment	Before treatment	After treatment
Observation group (*n* = 36)	3.11 ± 1.47	1.68 ± 0.95^a^	3.39 ± 1.06	1.86 ± 0.96^a^	20.58 ± 2.07	10.84 ± 1.11^a^	3.05 ± 1.04	4.90 ± 1.24^a^	3.79 ± 1.31	5.81 ± 1.14^a^	41.15 ± 7.74	49.51 ± 4.63^a^
Control group (*n* = 36)	3.05 ± 0.87	2.20 ± 0.59^a^	3.68 ± 0.92	2.61 ± 0.75^a^	20.52 ± 3.73	12.07 ± 1.61^a^	3.02 ± 1.00	4.04 ± 0.94^a^	3.33 ± 0.85	4.80 ± 0.88^a^	42.01 ± 3.27	45.81 ± 2.78^a^
*t*	0.242	2.750	1.239	3.662	0.390	3.784	0.148	3.339	1.782	4.007	0.610	4.189
*P*	0.809	0.008	0.220	<0.001	0.698	<0.001	0.883	0.001	0.079	<0.001	0.544	<0.001

Note: compared with before treatment, ^a^*P* < 0.05.

**Table 4:** Comparison of pain and function scores between the two groups (^−^*x* ± *s*, points).

Group	VAS score		BASDAI score		BASFI score	
	Before treatment	After treatment	Before treatment	After treatment	Before treatment	After treatment
Observation group (*n* = 36)	8.22 ± 0.68	4.64 ± 0.76^a^	26.67 ± 2.20	8.33 ± 1.20^a^	35.56 ± 3.84	9.22 ± 0.90^a^
Control group (*n* = 36)	8.14 ± 0.64	6.42 ± 0.65^a^	26.14 ± 2.80	15.00 ± 1.49^a^	35.14 ± 3.07	17.17 ± 1.13^a^
*t*	0.535	10.658	0.889	20.917	0.508	32.955
*P*	0.594	<0.001	0.377	<0.001	0.613	<0.001

Note: compared with before treatment, ^a^*P* < 0.05.

**Table 5:** Comparison of serum CXCL16, TNF-*α*, and IL-17 levels between the two groups (^−^*x* ± *s*).

Group	CXCL16 (g/l)		TNF-*α* (ng/l)		IL-17 (ng/l)	
	Before treatment	After treatment	Before treatment	After treatment	Before treatment	After treatment
Observation group (*n* = 36)	18.44 ± 3.67	10.05 ± 1.22^a^	41.91 ± 4.74	25.23 ± 3.35^a^	33.16 ± 3.67	18.98 ± 1.38^a^
Control group (*n* = 36)	18.88 ± 2.71	14.68 ± 1.50^a^	41.94 ± 4.98	32.80 ± 3.04^a^	33.19 ± 3.36	25.76 ± 2.16^a^
*t*	0.578	14.375	0.026	10.035	0.038	15.857
*P*	0.565	<0.001	0.979	<0.001	0.970	<0.001

Note: compared with before treatment, ^a^*P* < 0.05.

**Table 6:** Comparison of serum DKK-1, SOST, and BMP-2 levels between the two groups (^−^*x* ± *s*).

Group	DKK-1 (ng/l)		SOST (pg/ml)		BMP-2 (ng/l)	
	Before treatment	After treatment	Before treatment	After treatment	Before treatment	After treatment
Observation group (*n* = 36)	1678.01 ± 181.26	1392.82 ± 124.19^a^	50.76 ± 7.07	72.32 ± 6.62^a^	258.58 ± 25.45	158.12 ± 15.19^a^
Control group (*n* = 36)	1672.98 ± 139.39	1468.51 ± 161.22^a^	50.19 ± 5.14	64.02 ± 5.32^a^	257.51 ± 27.84	192.19 ± 19.03^a^
*t*	0.132	2.231	0.387	5.864	0.171	8.396
*P*	0.895	0.029	0.700	<0.001	0.864	<0.001

Note: compared with before treatment, ^a^*P* < 0.05.

**Table 7:** Comparison of drug safety between the two groups (cases (%)).

Group	Nausea	Ventosity	Sour regurgitation	Rash	WBC decline	ALT rise	Total adverse reaction
Observation group (*n* = 36)	1 (2.78)	1 (2.78)	0 (0.00)	2 (5.56)	1 (2.78)	1 (2.78)	6 (16.67)
Control group (*n* = 36)	0 (0.00)	1 (2.78)	1 (2.78)	1 (2.78)	0 (0.00)	0 (0.00)	3 (8.33)
Fisher exact probability							0.478

## Data Availability

The labeled dataset used to support the findings of this study are available from the corresponding author upon request.

## References

[1] Soulard J., Vaillant J., Agier C. T., Vuillerme N. (2021). Gait characteristics in patients with ankylosing spondylitis: a systematic review. *Clinical and Experimental Rheumatology*.

[2] Benucci M., Damiani A., Bandinelli F., Grossi V., Atzeni F. (2018). Ankylosing spondylitis treatment after first anti-TNF drug failure. *The Israel Medical Association Journal*.

[3] Zhang P., Zhou S., Chen Z., Tian Y., Guo C. (2021). TNF receptor: fc fusion protein downregulates RANKL/OPG ratio by inhibiting CXCL16/CXCR6 in active ankylosing spondylitis. *Current Pharmaceutical Biotechnology*.

[4] Ustun N., Tok F., Kalyoncu U., Motor S., Turhanoglu A. (2014). Sclerostin and Dkk-1 in patients with ankylosing spondylitis. *Acta Reumatológica Portuguesa*.

[5] Chisălău B. A., Crînguș L. I., Vreju F. A. (2020). New insights into IL-17/IL-23 signaling in ankylosing spondylitis (review). *Experimental and Therapeutic Medicine*.

[6] Van der Linden S., Valkenburg H. A., Cats A. (1984). Evaluation of diagnostic criteria for ankylosing spondylitis. *Arthritis & Rheumatism*.

[7] Zheng X. Y. (2002). *Guidelines for Clinical Research of New Chinese Medicines*.

[8] Wang T. F., Yang Y. L., Xue X. L. (2012). *Traditional Chinese Medicine Diagnostics*.

[9] Sun B., Che X. M. (2012). Visual analogue scale (VAS). *Chinese Journal of Neurosurgery*.

[10] Song J., Zhou L., Chen L., Wu X., Xu H. (2015). Comparison of disease activity indicators ASDAS, RAPID3 and BASDAI in judging disease activity in patients with ankylosing spondylitis. *Journal of the Second Military Medical University*.

[11] Wen Q. F., Yang J. S., Ji X. J. (2016). The application value of SF-36 scale and clinical evaluation index in ankylosing spondylitis cohort study. *Chinese Medical Journal*.

[12] Li S., Li R., Zeng Y., Meng X. L., Wen C. B., Zheng S. C. (2019). Chemical components and pharmacological action of Aconiti Radix. *Zhongguo Zhong Yao Za Zhi*.

[13] Xia T., Dong X., Jiang Y. (2019). Metabolomics profiling reveals Rehmanniae Radix Preparata extract protects against glucocorticoid-induced osteoporosis mainly via intervening steroid hormone biosynthesis. *Molecules*.

[14] Zuo Z. Y., Zhan S. Y., Huang X., Ding B. Y., Jiang N. H. (2017). Research progress of pharmacokinetics and pharmacodynamics of total glucosides of peony in hepatoprotective effects. *Zhongguo Zhong Yao Za Zhi*.

[15] Wang X. M., Xu L. K., Luo J. B. (2020). Study on the anti-inflammatory and analgesic effects of Ephedra and Guizhi. *New Chinese Medicine and Clinical Pharmacology*.

[16] Wang Z., Wang D., Yang D., Zhen W., Zhang J., Peng S. (2018). The effect of icariin on bone metabolism and its potential clinical application. *Osteoporosis International*.

[17] Hu N., Wang C. H., Wang B. H. (2022). Qianghuo Shengshi decoction exerts anti-inflammatory and analgesic via MAPKs/CREB signaling pathway. *Journal of Ethnopharmacology*.

[18] Guo F. F., Tang X., Tang L. Y., Wei J. Y., Xiao J. P., Yang H. J. (2020). Comparative study on the efficacy and material basis of different parts of Eucommia ulmoides based on network pharmacology. *China Journal of Traditional Chinese Medicine*.

[19] Wang X. L., Wu Y., Jiang S. H., Hu L. W., Ping L. F. (2018). Clinical study of Tongbi capsule in the treatment of knee osteoarthritis caused by cold dampness. *Shaanxi Traditional Chinese Medicine*.

[20] Mo J. F., Bao Y., Ruan L. J., Ye Q. (2019). Expression and mechanism of CXC chemokine ligand 16 in ankylosing spondylitis. *Chinese Journal of Experimental Surgery*.

[21] Pedersen S. J., Maksymowych W. P. (2019). The pathogenesis of ankylosing spondylitis: an update. *Current Rheumatology Reports*.

[22] Tsukazaki H., Kaito T. (2020). The role of the IL-23/IL-17 pathway in the pathogenesis of spondyloarthritis. *International Journal of Molecular Sciences*.

[23] Liao H. T., Lin Y. F., Tsai C. Y., Chou T. C. (2018). Bone morphogenetic proteins and Dickkopf-1 in ankylosing spondylitis. *Scandinavian Journal of Rheumatology*.

[24] Sun W., Tian L., Jiang L. (2019). Sclerostin rather than Dickkopf-1 is associated with mSASSS but not with disease activity score in patients with ankylosing spondylitis. *Clinical Rheumatology*.

[25] Wang G., Cai J., Zhang J., Li C. (2018). Mechanism of triptolide in treating ankylosing spondylitis through the anti-ossification effect of the BMP/Smad signaling pathway. *Molecular Medicine Reports*.

